# Cortical thickness and its associations with age, total cognition and education across the adult lifespan

**DOI:** 10.1371/journal.pone.0230298

**Published:** 2020-03-25

**Authors:** Christian Habeck, Yunglin Gazes, Qolamreza Razlighi, Yaakov Stern

**Affiliations:** Cognitive Neuroscience Division, Department of Neurology, Columbia University Medical Center, New York, NY, United States of America; Nathan S Kline Institute, UNITED STATES

## Abstract

Early-life education (years of schooling) has been investigated in regards to cognition, health outcomes and mortality. It has been shown to confer cognitive reserve that might lessen the impact of brain pathology and its impact on cognitive and motor functioning in a variety of neurodegenerative diseases and, for instance, to influence electrical activity [Begum, T., Reza, F., Ahmed, I., & Abdullah, J. M. (2014). Influence of education level on design-induced N170 and P300 components of event related potentials in the human brain. *J Integr Neurosci*, *13*(1), 71–88. doi:10.1142/S0219635214500058]. On the other hand, demonstrations of a direct association between education and brain-structural measures have been more equivocal and scant. The current study sought to identify univariate cortical-thickness patterns underlying education and general intelligence after adjusting for age, gender and possible in-scanner movement in 353 individuals aged 40 to 80. We followed up this idea with multivariate analyses as well. For univariate analyses, our analyses yielded no robust associations between education and general intelligence beyond confounding effects of gender, age and extraneous in-scanner movement. A subsequent multivariate analyses showed a relationship between education and regional cortical thickness with a robust pattern of negative as well as positive loadings in several right-sided brain areas, speaking to a subtle but robust distributed effect of education on cortical thickness. Cortical thickness variance that is the residual of this education-related pattern was shown to be positively associated with age and extraneous in-scanner movement. Our study thus presents a complex picture of the association of education with regional cortical thickness: education was associated with a distributed brain-wide pattern of positive as well as negative loadings with unaccounted residuals being larger for older participants. Focal regional associations beyond demographic and age covariates were not identified.

## Introduction

Education is a major influence in childhood and early adulthood, with repercussions on occupational and socioeconomic outcomes throughout the adult life span. Intelligence, on the other hand, is a factor that partly results from the influence of education, innate talent driven by genetics, and brain structure. Associations between cortical thickness and intelligence have been identified in a variety of study settings and samples. Young adults show clear regional thickness-intelligence associations cross-sectionally [1], while a life-span sample demonstrated that thickness-intelligence relationships are not time-invariant across the life span, with a reversal of thickness-intelligence relationships around young middle age in a longitudinal data set [2]. In addition to the quest for group-level structural thickness patterns underlying intelligence, several studies also show a clear link of omnibus brain measures (like global cortical thickness and volume) to intelligence [3] as well as a relationship between higher-order regional thickness features (within-region variance in addition to mean) and intelligence [4].

For education, there are few cross-sectional studies; findings regarding the correlation with thickness are mixed, with both supporting evidence of correlations in areas associated with Alzheimer-related cortical thinning [5,6] but also lack of confirmation of correlations in studies with larger sample sizes [7]. An interesting analysis on life-span data [8] found that cortical thickness at age 73 was correlated with education, but that this association lessened significantly when childhood intelligence at age 11 was entered into the model, hinting at possible over-estimations of pure education-related associations. In addition to inconsistent direct associations between education and cortical thickness, interactions with factors such as exercise have been noted [9]. Very few studies have examined the direct effect of an education *intervention* on cortical thickness [10] and such studies usually possess only small sample sizes, but education level has been demonstrated to be related to better brain maintenance, i.e. reduced age-related atrophy, and cognitive reserve, but the studies have not been unequivocal [11,12]

Both intelligence and educations thickness relations are dwarfed by associations with age and ageing, e.g. [13–17]. The current study aimed to systematically investigate the association of education with cortical thickness and contrast it to the association with intelligence, carefully controlling for chronological age. Intelligence was operationalized as the composite of cognitive performance in 4 cognitive domains: (1) episodic memory, (2) reasoning ability, (3) perceptual speed, and (4) vocabulary. We performed standard region-wise analyses for associations between cortical thickness with total cognition and education, and for an association of the variability across participants in cortical thickness with education and total cognition.

Finally, to allow for the possibility that associations with education or total cognition cannot be localized robustly to key areas, we sought to identify cortical-thickness patterns which might hint at more distributed effects with multivariate analysis. Identification of multivariate patterns underlying education or total cognition allows an inspection of residual cortical thickness maps unaccounted for by the thickness patterns, and how such residuals are associated with chronological age.

## Methods

### Participant sample

We list the main characteristics of our sample below, broken down by age. All procedures were approved by the local Columbia University Medical Center Institutional Review Board; informed consent was obtained from all participants.

Participants were recruited via random-market-mailing, and screened for MRI contraindications and hearing or visual impairment that would impede testing. Older adult participants were screened for dementia and mild cognitive impairment prior to participating in the study, and participants who met criteria for either were excluded. Apart from these cognitive exclusion criteria, there were other health-related exclusion criteria including: myocardial infarction; congestive heart failure or any other heart disease; brain disorder such as stroke, tumor, infection, epilepsy, multiple sclerosis, degenerative diseases; head injury (loss of consciousness > 5mins); intellectual disability; seizure; Parkinson’s disease; Huntington’s disease; normal pressure hydrocephalus; essential/familial tremor; Down Syndrome; HIV Infection or AIDS diagnosis; learning disability/dyslexia; ADHD or ADD; uncontrolled hypertension; uncontrolled diabetes mellitus; uncontrolled thyroid or other endocrine disease; uncorrectable vision; color blindness; uncorrectable hearing and implant; pregnancy; lactating; any medication targeting central nervous system; cancer within last five years; renal insufficiency; untreated neurosyphillis; any alcohol and drug abuse within last 12 months; recent non-skin neoplastic disease or melanoma; active hepatic disease; insulin dependent diabetes; any history of psychosis or ECT; recent (past 5 years) major depressive; bipolar, or anxiety disorder; objective cognitive impairment (dementia rating scale of <130); and subjective functional impairment (BFAS > 1). The prevalence of medication for hypertension, diabetes, and high cholesterol is, respectively: 18%, 14%, and 7%. This compares favorably with CDC statistics for the adult US population at large (33.5%, 12.6%, and 12.1%, from www.cdc.gov/nchs/fastats). A complete description of the participants in terms of demographics and cortical thickness can be found in Table 1.

**Table 1:** Sample characteristics, broken down by age decade. NARTIQ = North American Reading Test for adults [18], DRS = Dementia Rating Scale [19].

	**All**	**40–49**	**50–59**	**60–69**	**>70**
**N**	**353**	**43**	**67**	**167**	**76**
**NART-IQ**	**118 ± 9**	**114 ± 8**	**116 ± 9**	**119 ± 8**	**120 ± 8**
**Education**	**16.3 ± 2.4**	**16.1 ± 2.6**	**16.0 ± 2.0**	**16.2 ± 2.3**	**16.8 ± 2.6**
**Gender**	**191F, 162M**	**18F, 25M**	**34F, 33M**	**93F, 74M**	**46F, 30M**
**DRS**	**140.0 ± 2.8**	**139.9 ± 2.8**	**139.9 ± 2.5**	**139.5 ± 2.9**	**140.1 ± 2.8**
**Mean Cortical thickness**	**2.57 ± 0.11**	**2.65 ± 0.37**	**2.60 ± 0.39**	**2.56 ± 0.37**	**2.51 ± 0.35**

### Assessment of total cognition

Four domains of cognitive functioning were assessed with three tasks each. A summary score was calculated for each domain by averaging the z-scores of the three tasks under each domain.

### Memory

Three sub-scores of the Selective Reminding Task (SRT) [20] were selected. Participants in this task were initially read a list of 12 words and asked to recall as many as they could. For the following five trials they were reminded of the words that they did not report and were asked to again recall all of the words in the list. Words are considered to enter long term storage from the point when they are recalled twice in a row without reminders. The long-term storage sub-score (SRTLTS) is the sum over all words of the number of trials when each word was in long-term storage. Continuous long-term retrieval (SRT CLRT) is the sum over all words of the number of trials for which the word was continuously recalled. The third memory measure was the number of words recalled on the last trial (SRT Last).

### Perceptual speed

One selected measure was the score on the Digit Symbol subtest from the Wechsler Adult Intelligence Scale (WAIS III) [21]. Participants in this test were instructed to write the symbol corresponding to specific numbers as quickly as possible based on a key specifying the appropriate symbol for each digit. The score is the number of correctly produced symbols in 90 seconds. A second measure was the score on Part A of the Trail Making Test [22], in which participants are instructed to connect circles numbered from 1 to 24 as rapidly as possible and performance is assessed as the time to connect all 24 circles. The third speed measure was the number of colored ink patches named in 45 seconds in the Stroop Color Naming test.

### Reasoning ability

One test was the WAIS III [21] Block Design test, in which participants are asked to reproduce a series of increasingly complex geometrical shapes using 4 or 9 identical blocks with red, white, or split red and white sides. A second test was the WAIS III [19] Letter-Number Sequencing test in which participants are asked to recall progressively longer lists of intermixed letters and numbers in alphabetical and then numerical order. The third reasoning test was the Ravens Progressive Matrices test [23] in which participants are asked to select which pattern in a set of eight possible patterns best completes a missing cell in a matrix.

### Vocabulary

Tasks included the Vocabulary subtest from the WAIS III [21], the Wechsler Test of Adult Reading (WTAR) [21], and the American National Adult Reading Test (AMNART) [24]. The Vocabulary subtest asks participants to provide definitions for a series of increasingly advanced words, and the WTAR and AMNART both involve participants correctly pronouncing irregularly spelled English words.

Z-scores for each of the cognitive tests were calculated, and if necessary sign-reversed, such that higher scores implied better cognitive performance. All Z-scores were then averaged to create a composite Z-score, which was used as our total-cognition score in this study.

### Structural brain data acquisition

All scans were acquired on a 3.0 Tesla Philips Achieva MRI scanner. A T1-weighed (MPRAGE) scan was used. The scans were acquired with TE/TR of 3/6.5 ms and Flip Angle of 8 degrees, in-plane resolution of 256 x 256, field of view of 25.4 x 25.4 cm, and 165–180 slices in axial direction with slice-thickness/gap of 1/0 mm. The FreeSurfer (v5.1.0) software for human brain imaging analysis (http://surfer.nmr.mgh.harvard.edu/) was used for the reconstruction of the T1 scans [25,26] and computation of average cortical thickness in 68 native-space Regions Of Interest (ROIs) [27]. Every structural scan was visually inspected to ensure good FreeSurfer performance.

### Association with subject motion

Due to recent reports about possible motion confounds even in structural neuroimaging data [28] we located any possible functional MRI scans with available attendant realignment parameters. The number of task-runs (including resting state) for which mean relative frame-wise displacement was available ranged from 6 to 109. We computed the mean relative subject frame-wise displacement rFD, across volume in a run, and then across runs, and used it as a covariate of no interest in our analyses.

We computed the bivariate correlations between all our subject variables, i.e. education, total cognition, gender, relative frame-wise displacement, and age.

The table shows collinearity between some of the variables as expected. After adjusting for all other covariates in partial correlations, we found age to correlate negatively with total cognition, but positively with education. Education correlated positively with cognition, and in-scanner movement correlated negatively with cognition. The associations between age, cognition and education were found to *strengthen* after partial correlations, suggesting strong collinearities, and the need for simultaneous adjustment in both our univariate and multivariate analyses in this paper.

### Differential thickness associations between age, cognition, and education

First, we established associations between cortical thickness on the one hand, and age, education, and total cognition on the other hand. To this end, we ran a region-wise regression model

Corticalthickness(i)=[educationgendercognitionrFDage]β(i)+εi=1…68

where all variables are column vectors and **β** is the 5-component vector of regression weights. We looked to all regression weights, with particular emphasis on education and total cognition, and identified regions associated with each variable at a False Discovery Rate (FDR) [29] of q = 0.05.

We also ran a single brain-behavioral model for mean cortical thickness.

### Regional variance analyses

In addition to the region-wise brain-behavioral models, we were also interested whether the inter-subject variance in cortical thickness showed significant relationships with education or total cognition. This we residualized the regional cortical thickness data with respect to all covariates apart from our covariate of interest (education, total cognition). After performing a median split in the covariate of interest, we compute a regional log-F statistic as

log‑F(i)=log[rVAR(i;HIGHcovariatevalue)/rVAR(i;LOWcovariatevalue)]i=1…68

where rVAR (i; LOW), for instance, denotes the inter-subject variance in residual cortical thickness in region *i* across all participants who fall below the median-split value of the covariate of interest.

For an inferential judgment of statistical significance, we than ran a permutation test with 10,000 where the assignment between brain and subject variables was randomized. The computation of residualization and log-F statistic ensued each time, producing a null-histogram on which to base a two-tailed test of significance.

We show an example for clarity below in Fig 1, where the residualized cortical-thickness in the left pars opercularis is shown to be *lower* for participants with *higher* total cognition.

**Fig 1:** Non-parametric permutation F-test with 10,000 iterations for the residualized thickness variance with respect to total cognition. In this region, the left pars opercularis, higher total cognition is associated with *lower* thickness variance at p = 0.0129 (uncorrected for multiple comparisons). The point estimate for the log-F statistic is shown with a thin black line in the left tail of the null-distribution.

### Adjusted multivariate PCA-regression to derive an education-related cortical-thickness pattern

In addition to the univariate analyses, we also decided to perform multivariate analyses with a similar adjustment to account for the collinearities in the 5 subject variables shown before. If we assume an N x 4 array of confounding variables called **C** (comprising total cognition, gender, rFD and age) we can apply some simple matrix algebra to effect such residualization. The influence of the confounders will be removed from both thickness array as well as the dependent variable, education, prior to performing a multivariate PCA-regression. For the following explanations, we only used education as the dependent variable, and total cognition was one of the covariates. However, we also switched the roles of education and total cognition, and tried to derive an adjusted thickness pattern related to total cognition. However, no significant results were identified, and for clarity we adopted education as the dependent variable for the following explanation.

For education residualization is written with a projection operator as:

$$rEdu=\left(1–C\;{\left(C\;C\right)}^{‐1}\;C\right)\;DV$$

where **1** denotes the 353 x 353 unit matrix (given that there are 353 participants in our study). The same projection works for the subject scores of all Principal Components. We can write the cortical-thickness data array, **THX**, as the product of Principal Components in **V** and subject scores in **W,**

THX=VW,[THX]=68x353,[V]=68x67,[W]=353x67

where [] denotes the matrix dimensions and ‘ implies matrix transposition. Because we removed the grand-mean image from the thickness data, we only have 67 = 68–1 Principal Components. We can now apply the projection operator simultaneously to all columns of **W** as

$$rW=(1–C\;{\left(C\;C\right)}^{‐1}\;C)\;W.$$

After multiplication from the right with the Principal Component array, r**THX** = **V** r**W**, we have created a (residualized) thickness array that is independent of linear effects of all nuisance variables in **C**. **rTHX** has the same format as **THX,** and can be subjected to PCA-regression (explained in the following section) to derive a pattern related to r**Edu**.

After the residualization computations, we are ready to apply a well-honed and simple multivariate technique, the Scaled Subprofile Model, a form of PCA-regression [30–32] to our residualized thickness array to derive patterns whose expression best predicts the residualized dependent variable.

Briefly, we reran PCA, but this time on the residualized data, **rTHX**, and obtained an array of K Principal Components in **V.** The subsequent regression is performed according to:

rEdu=[rTHXV1]β+ε

In short, we projected a set of Principal Components into the thickness data to obtain subject scores of all PCs, and then performed a linear regression with the outcome of interest (= education or total cognition) as the dependent variable. The set of selected Principal Components 1:K in **V** was chosen via leave-one-out cross-validation to minimize the predicted residual sum of squares (= PRESS). A corresponding cortical-thickness pattern can then be constructed according to

v=Vβ(1:K).

This pattern assigns loadings to each of the 68 ROIs. The loadings are normalized such that squaring and summing them yields unity, or written with the L-2 norm: L(**v**,2) = 1. This normalization implies that all variance information is carried in the subject pattern score, which can be obtained according to the projection

w=rTHXv

and is column vector with as many rows as participants.

To get an idea of the inferential robustness of these loadings, we performed the whole analytic recipe, PCA with subsequent brain-behavioral regression after repeatedly sampling with replacement from r**Edu** and r**THX** in a bootstrap procedure [33] with 10,000 iterations. Regions with robust loadings in the pattern were identified as having the [2.5% 97.5%] coverage interval across the 10,000 iterations outside of the zero point.

The last thing in our multivariate analysis is to see whether residual signal *not* accounted for by the derived pattern relates to any of the covariates. We can write our data array with the pattern score vector, **w**, and the pattern, **v**, as

rTHX=vw+Ε

where **Ε** denotes the residual signal not captured by the education-related thickness pattern, and has the dimensions

[Ε]=68x353.

We can square this data array, transpose it and average the squared values across regions arrive at a 353 x 1 column vector of subject-wise residual sum of squares as indicated with this Matlab notation:

RESS=mean(E.^2,1).

This vector serves as a dependent variable in a regression against our covariates to find out whether and how the covariates are related to the amount of residual activity orthogonal to the educated-related thickness patterns. Positive relationships, for instance with age, would imply that for older people the amount of thickness variance *not* captured by the pattern is higher than for younger people.

We display toy example to demonstrate the concept of residual signals. We emphasize that the data displayed in Fig 2 are simulated and not real. For simplification we assume that we only have 2 ROIs (instead of 68) which permits visualization in a simple scatter plot. A brain thickness map can be seen as a point with (x,y) in a 2-d coordinate system. Our covariance pattern was assumed to be **v** = [1;1]/sqrt(2). Variance associated with this pattern can be seen as a straight line with slope = 1 in this simple example. Residual signal with respect to **v** can be seen as the shortest distances of any point (x,y) to the line. (In contrast to a standard regression line y = f(x), the residuals are *not* just the vertical offsets, which would only quantify the difference between predicted and actual y-values. The multivariate residuals consider all dimensions.)

**Fig 2:** Explanation of residual signal not accounted for by a multivariate thickness pattern. The figure shows a toy example with 2 ROIs (ROI1 = x-coordinate, ROI2 = y-coordinate), and every data point can be represented by a duplet (x,y). Residual activity with regard to the covariance pattern **v** = [1;1]/sqrt(2) can be understood as the squared shortest distance of every point (x,y) with regard to the straight line y = x.

Again, we will assess whether there is structure in these residuals according to the regression

RESS=[educationgendercognitionrFDage]β+ε.

A positive association, for instance, between **RESS** and age would be imply that the education-related thickness pattern accounts for less variance in the thickness data for older people as residual signal becomes more prominent.

## Results

### Association of cortical thickness with covariates

We first conducted ROI-wise regression analysis (Eq.1), and then performed FDR corrections for multiple comparison with Q<0.05. The results of all brain-behavioral regressions are displayed in Table 2. No significant associations were found between regional cortical thickness and education or total cognition at Q<0.05. Significant associations were found for the other covariates however. (See Table 2). Gender was related to cortical thickness in 27 regions, and for 26 of those, women showed higher cortical thickness than men. In-scanner movement obtained from any available functional scans as mean relative frame-wise displacement was related negatively to cortical thickness in 9 regions. Age correlated with cortical thickness in 62 regions in a negative direction, as expected.

**Table 2:** FDR-corrected associations (Q<0.05) between regional thickness and gender, rFD and age, from multiple linear regressions with education, total cognition, gender, rFD, and age as simultaneous, z-standardized, covariates. No associations at Q<0.05 were found for education and total cognition.

FS regional label	T	β	Uncorrected p
**Covariate: Gender, 27 regions**			
rh-frontalpole	4.3065	0.0690	2.1619e-05
rh-rostralmiddlefrontal	4.1324	0.0306	4.505e-05
rh-lateraloccipital	4.1315	0.0304	4.5225e-05
rh-superiorfrontal	4.0727	0.0300	5.7616e-05
lh-lateraloccipital	4.0664	0.0287	5.9115e-05
lh-inferiorparietal	3.7874	0.0266	0.0001794
rh-isthmuscingulate	3.7164	0.0412	0.00023548
rh-postcentral	3.6077	0.0247	0.00035432
lh-superiorfrontal	3.6074	0.0249	0.00035467
rh-inferiorparietal	3.5902	0.0251	0.00037798
rh-posteriorcingulate	3.5812	0.0345	0.00039077
lh-postcentral	3.5744	0.0251	0.00040079
lh-paracentral	3.4547	0.0298	0.00061921
lh-supramarginal	3.1780	0.0214	0.0016163
rh-paracentral	3.1085	0.0269	0.0020359
lh-middletemporal	3.1019	0.0246	0.0020804
rh-parahippocampal	2.9900	0.0453	0.0029888
lh-parsorbitalis	2.9598	0.0333	0.0032896
lh-rostralmiddlefrontal	2.9534	0.0216	0.0033572
lh-parahippocampal	2.8365	0.0500	0.0048285
rh-parsorbitalis	2.7826	0.0317	0.0056869
lh-isthmuscingulate	2.7048	0.0295	0.0071706
lh-entorhinal	-2.6344	-0.0596	0.0088054
lh-pericalcarine	2.5495	0.0246	0.011217
rh-superiorparietal	2.4661	0.0177	0.014142
rh-precentral	2.4287	0.0177	0.015661
lh-frontalpole	2.3485	0.0382	0.019412
**Covariate: rFD, 10 regions**			
rh-lateralorbitofrontal	-4.6001	-0.0448	5.9281e-06
rh-medialorbitofrontal	-4.5305	-0.0473	8.105e-06
lh-insula	-3.7699	-0.0331	0.00019192
rh-entorhinal	-3.4029	-0.0808	0.00074476
lh-temporalpole	-3.3097	-0.0715	0.0010321
lh-superiorparietal	-2.9854	-0.0225	0.0030331
lh-lateralorbitofrontal	-2.9370	-0.0274	0.0035355
rh-inferiortemporal	-2.9214	-0.0268	0.0037124
rh-insula	-2.8468	-0.0273	0.0046786
rh-temporalpole	-2.7141	-0.0665	0.0070
**Covariate: Age, 62 regions**			
rh-superiortemporal	-8.7436	-0.0785	9.8729e-17
lh-superiortemporal	-8.2074	-0.0686	4.4823e-15
rh-parstriangularis	-7.8860	-0.0737	4.0954e-14
lh-superiorfrontal	-7.8802	-0.0567	4.2606e-14
lh-middletemporal	-7.7075	-0.0639	1.3632e-13
lh-parstriangularis	-7.5693	-0.0673	3.4181e-13
lh-parsopercularis	-7.4748	-0.0568	6.3601e-13
lh-parsorbitalis	-7.3592	-0.0865	1.3507e-12
lh-inferiorparietal	-7.1970	-0.0528	3.8317e-12
rh-middletemporal	-7.0475	-0.0588	9.8743e-12
rh-bankssts	-7.0151	-0.0686	1.21e-11
lh-bankssts	-6.7806	-0.0640	5.1655e-11
lh-precuneus	-6.7788	-0.0486	5.2205e-11
rh-parsopercularis	-6.5617	-0.0548	1.9367e-10
rh-precuneus	-6.5160	-0.0462	2.542e-10
rh-superiorfrontal	-6.4274	-0.0494	4.2895e-10
lh-supramarginal	-6.3562	-0.0446	6.5088e-10
rh-supramarginal	-6.1671	-0.0456	1.935e-09
lh-lateralorbitofrontal	-5.8496	-0.0558	1.1396e-08
rh-parsorbitalis	-5.7864	-0.0688	1.6079e-08
lh-precentral	-5.7830	-0.0425	1.6378e-08
rh-lateralorbitofrontal	-5.7624	-0.0575	1.8309e-08
rh-precentral	-5.6964	-0.0434	2.6122e-08
rh-fusiform	-5.5166	-0.0477	6.7675e-08
lh-isthmuscingulate	-5.3839	-0.0613	1.3454e-07
lh-fusiform	-5.2926	-0.0449	2.1423e-07
rh-inferiortemporal	-5.2921	-0.0497	2.1477e-07
rh-inferiorparietal	-5.2213	-0.0381	3.068e-07
rh-rostralmiddlefrontal	-5.1206	-0.0395	5.0586e-07
rh-medialorbitofrontal	-4.6703	-0.0499	4.3062e-06
lh-paracentral	-4.4352	-0.0399	1.2365e-05
lh-insula	-4.4280	-0.0398	1.2762e-05
lh-medialorbitofrontal	-4.4190	-0.0442	1.3274e-05
rh-frontalpole	-4.4086	-0.0738	1.3894e-05
rh-paracentral	-4.3660	-0.0395	1.672e-05
rh-lateraloccipital	-4.3153	-0.0331	2.081e-05
lh-inferiortemporal	-4.2581	-0.0400	2.6575e-05
lh-superiorparietal	-4.2195	-0.0326	3.1295e-05
rh-lingual	-4.1593	-0.0339	4.0277e-05
lh-transversetemporal	-3.9760	-0.0454	8.5317e-05
lh-lateraloccipital	-3.8292	-0.0282	0.00015251
lh-rostralmiddlefrontal	-3.6255	-0.0276	0.00033157
rh-caudalmiddlefrontal	-3.5971	-0.0291	0.00036848
lh-posteriorcingulate	-3.4777	-0.0337	0.00057011
lh-temporalpole	-3.3103	-0.0732	0.0010298
rh-superiorparietal	-3.2969	-0.0247	0.0010785
lh-postcentral	-3.2396	-0.0238	0.0013125
lh-caudalmiddlefrontal	-3.1997	-0.0235	0.0015027
lh-frontalpole	-3.1167	-0.0529	0.0019813
rh-postcentral	-3.1104	-0.0222	0.0020233
lh-rostralanteriorcingulate	-2.8486	-0.0342	0.0046538
rh-cuneus	-2.6593	-0.0223	0.0081926
rh-isthmuscingulate	-2.6503	-0.0307	0.0084108
rh-temporalpole	-2.6284	-0.0659	0.0089599
rh-rostralanteriorcingulate	-2.4503	-0.0287	0.014769
rh-insula	-2.2881	-0.0225	0.022734
lh-parahippocampal	-2.2004	-0.0405	0.028434
rh-entorhinal	-2.1295	-0.0518	0.033915
rh-pericalcarine	-2.1144	-0.0178	0.035192
rh-posteriorcingulate	-2.0831	-0.0209	0.03797
lh-entorhinal	-2.0285	-0.0479	0.043276
lh-lingual	-2.0210	-0.0192	0.044044

When regressing mean cortical thickness in the regression model, significant effects at p<0.05 were found for all covariates apart from education (total cognition: T = 2.2424, p = 0.0256; gender: T = 2.6532, p = 0.0083; rFD: T = -3.1160, p = 0.0020; age: T = -7.7074, p<0.0001). Better total cognition and being female are thus associated with higher mean thickness, while higher in-scanner movement and age are associated with lower thickness.

### Variance of cortical thickness in regard to education and total cognition

We performed non-parametric permutation F-test to check whether adjusted residual cortical variance displays *higher* or *lower* inter-subject variance for subjects above the median split in either education or total cognition. No regional test surpassed the FDR threshold of Q<0.05 for either education or total cognition.

### Multivariate education-related thickness pattern

Applying our adjusted multivariate PCA-regression to derive a thickness pattern related to total cognition did not succeed. The leave-one-out cross-validation procedure retrieved PCs 1–3 as the best-fitting set, but the brain-behavioral regression was not significant at p = 0.1912.

The same analytic recipe, however, produced a significant finding for education: PCs 1–4 were used to construct a pattern whose subject scores correlated with residualized education at R = 0.1898, p = 0.0123. (By construction, the correlation with all other covariates was R = 0.) The results of the cross-validation procedure and brain-behavioral correlation pertaining to the pattern can be seen in Fig 3.

**Fig 3:** Results of the adjusted multivariate analysis to derive an education-related cortical-thickness pattern. Panel A (left) shows the leave-one-out cross validation results which yield minimum mean PRESS for 4 Principal Components. Panel B (right) shows the relationship between subject scores of the derived pattern and the residualized education variable.

We also ran a bootstrap procedure with 10,000 iterations to find robust loadings whose [2.5% 97.5%] coverage interval does not include the zero point.

We could identify 4 regions, 2 with robust positive and 2 with robust negative loadings, respectively, all lateralized to the right side of the brain. Robust positive loadings were found for the right isthmus and anterior cingulate; robust negative loadings were found for the right superior temporal gyrus and temporal pole. The loadings are listed in Table 3, and the loading distributions are shown as line plots in Fig 4 for completeness.

**Fig 4:** 95% coverage intervals, i.e. from 2.5%ile to 97.5%ile, plotted for all regional loadings by bootstrap procedure with 10,000 iterations. Left panel: left-side side regions; right panel: right-side regions. The regions whose 95%-coverage intervals did not include the zero point were circled in gray color.

**Table 3:** Listing of the 4 regions that were identified with robust loadings in the bootstrap estimation procedure.

Region label	2.5% of bootstrap distribution	97.5% of bootstrap distribution
rh-isthmuscingulate +	0.0202	0.2469
rh-posteriorcingulate +	0.0016	0.2879
rh-superiortemporal -	-0.1218	-0.0008
rh-temporalpole -	-0.6854	-0.0099

Lastly, we computed the subject-wise residual sum of squares of thickness signal *not* captured by the covariance patters and regressed against all our covariates. The results are shown in Table 4.

**Table 4:** Linear regression of subject-wise residual sum of squares of thickness signal orthogonal to the derived education-related thickness pattern. In-scanner movement (= rFD) and age were associated positively with residual thickness signal.

Covariate	T	p-value
Education	0.2884	0.7732
Total cognition	-0.2132	0.8313
Gender	0.4296	0.6677
rFD	**4.1873**	**0.0000**
Age	**3.6859**	**0.0003**

Movement in the scanner and age were associated positively with residual cortical thickness that is not accounted for by the education-related pattern, while the remaining covariates showed no association.

## Discussion

We first give a summary of main findings with caveats about our study. In this study, we considered the group-level associations of education, age, gender, and total cognition with cortical thickness across middle and older age. Of particular interest were associations between education and total cognition on the one hand, and regional cortical thickness on the other hand.

After adjusting for the average movement in the scanner obtained from extraneous functional scans, gender and age, we could not identify significant associations between regional cortical thickness and total cognition or education. Age and in-scanner movement, however, were negatively related to regional cortical thickness. Being female was associated with higher cortical thickness. For the across-region mean of cortical thickness, we found a positive relationship with total cognition and being female, and a negative relationship with age and in-scanner movement; again, education proved elusive and did not manifest any relationship to mean cortical thickness.

We then investigated whether regional heteroscedasticity in cortical thickness was present with respect to education and total cognition. No significant findings for individual regions at q<0.05 or the total variance could be identified.

We then turned our attention to multivariate analysis to search for brain-wide distributed patterns underlying education and total cognition with adjusted PCA-regression where the influence of all confounders was removed from both brain data and dependent variable. We could identify a significant pattern for education, but not for total cognition. The pattern was localized on the right side and consisted of positive and negative loadings, indicating a relative thickening of positively loaded areas in the cingulate cortex, with a corresponding relative thinning of areas in the temporal cortex. We stress that due to the removal of the grand mean cortical-thickness pattern prior to the PCA, observations of lower and higher thickness with education are *relative* to the subject-wise overall mean thickness. This implies, that relative to their overall mean thickness, more educated participants had *larger* cortical thickness in right posterior and isthmus cingulate, but *lower* thickness in right superior temporal and temporal pole areas. These relative differences are correlated, i.e. the degree to which the positively loaded areas have relatively higher thickness is tightly linked to the degree to which the negatively loaded areas have lower thickness.

Due to the observational nature of the study, we cannot make causal statements, but an education-related thickening of positively loaded areas with a relative neglect of the negatively loaded areas would be consistent with our finding. The mechanism behind such a regional association of strengthening cortical thickness in select areas of the brain at the expense of other select areas is hard to conceive from the current vantage point.

Lastly, we inspected the residual sum of squares of subject thickness values *not* accounted for by (= orthogonal to) our derived pattern, and used it as a dependent variable in a linear regression with all our covariates as independent variables. Higher age and in-scanner movement in extraneous functional scans were associated with larger residual sum of squares, indicating that for older participants and participants who moved more during functional scans, the residuals to the relationship between education and cortical thickness were larger.

These results, obtained from quite involved computations, unfortunately are mainly null-findings, and failed to show regional associations of cortical thickness with total cognition and education. The only association of early-life education with cortical thickness in middle and older age was quite nuanced: cortices of longer educated people are thicker in right cingulate areas relative to right temporal areas.

When taking a step back and assessing our findings, we can say that they are not discordant with the prior literature since such direct cortical-thickness associations with education have been difficult to obtain[7]. Education is more often seen as an indirect influencing factor, for instance, for brain maintenance in the face of normal aging[5], neurodegenerative diseases such frontotemporal dementia [34], and Alzheimer’s [35]. Analyses aimed at establishing brain maintenance could only be performed as cross-sectional interactions between education and age on cortical thickness in our data: also here, we did not find anything that survived the FDR threshold.

We performed several additional unplanned analyses whose in-depth documentation would take up too much room and go beyond the scope of the paper. (1) We left out the in-scanner movement covariate to check whether this would unmask relationships between cortical thickness and our two covariates of interest (education, total cognition): no such relations were unmasked for education, but for total cognition several regions now survived the FDR-correction. (2) Further, we also performed region-wise mediation analysis [36] to check whether the effect of education on total cognition was mediated by regional cortical thickness: we only found mediation in the left parahippocampal gyrus, but it did not survive the FDR-correction.

## Conclusion

Our study showed that education to be associated with a distributed pattern of relatively larger thickness in right cingulate cortex, and a relatively lower thickness in right temporal areas, beyond confounding influences of age, total cognition and gender. Regional residual thickness variance that was orthogonal to this education-related pattern was shown to be larger for older people and people who moved more in extraneous functional scans.

Direct positive relationships between cortical thickness and either education or total cognition, on the other hand, even averaged across regions, could not be identified when taking into account a comprehensive array of confounding variables such as age, gender, and total cognition. In our study, age, education and total cognition had strong mutual associations, even after computing partial correlations (see Table 5). In light of these strong associations, maybe the difficulties in isolating a pure association between education and cortical thickness, unaffected by cognitive function, and vice versa, are not surprising.

**Table 5:** Relationships between all subject non-brain variables (= Pearson R). Bolded values denote statistical significance at p<0.05. The upper triangle lists partial correlations, the lower triangle unadjusted bivariate correlations. (rFD = Relative frame-wise displacement. Gender is coded as 1 = men, 2 = women).

	Education	Cognition	Gender	rFD	Age
Education	-	**0.35**	-0.04	-0.008	**0.21**
Cognition	**0.32**	-	-0.02	**-0.17**	**-0.26**
Gender	-0.05	-0.08	-	0.10	0.08
rFD	-0.07	**-0.22**	**0.12**	-	0.07
Age	**0.12**	**-0.23**	0.10	**0.12**	-

Trying to separate education from total cognition might require a substantial boost in statistical power. A better characterization of the content, rather than just the duration, of education will be necessary too. In our study, we estimate education to completed at least 10–15 years prior to the structural brain scan in middle and older age for all participants. Education as an “intervention” thus happened many years before the assessment of cortical thickness. The question remains whether the effects of education are such that regionally specific group-invariant associations can be uncovered at all, or whether boosted samples sizes are necessary to even identify associations of education with multimodal omnibus measures of structural brain health, i.e. which cannot be localized to particular brain regions or white-matter tracts. Education has shown to exert effects consistent with Cognitive Reserve [37–39], and be the putative cause of better cognition beyond individual brain-health endowments. Matching two individuals on all dimensions of brain measurement usually leaves any differences in cognition, at least partly, to be explained by education. The brain-structural substrates of education itself, on the other hand, are more difficult to identify and disentangle from cognition itself. These questions remain and form the basis for an exciting research program about the effects of education on the brain in the future.

## Supporting information

S1 File (XLSX)
